This article has been retracted.

# The Correlation and Copathogenesis of Coronary Aortic Sandwich and Renal Cysts

**DOI:** 10.1155/2022/5483155

**Published:** 2022-08-10

**Authors:** Huawei Zhang, Liang Gong, Zhinan Wu, Xuefen Luo

**Affiliations:** ^1^Longyan First Affiliated Hospital of Fujian Medical University, Cardiac and Vascular Surgery, Longyan 364000, Fujian, China; ^2^Longyan First Affiliated Hospital of Fujian Medical University, Ultrasonography Dept, Longyan 364000, Fujian, China

## Abstract

**Objective:**

To determine the correlation for aortic occlusion and hydronephrosis and the pathogenesis of copathogenesis.

**Methods:**

A retrospective census was established to probe the correlation with renal cysts by gathering aortic coarctation details concerning generic symptoms, diabetes, and liver and kidney profiles from 244 hospitalized aortic clinographers from April 2014 to December 2021 (study category, SG category), 150 hypertensive clients with primary hypertension attending our institution in the same period (matched category, MG category), and 150 able-bodied volunteers (control category, CG category).

**Results:**

(1) Intercategory discrepancies in regard to aortic occlusion, diabetic malfunction, and kidney and liver abnormality were neither mutually nor predominantly measured (*P* > 0.05); (2) 244 enrolled SG for aortic occlusion and 150 CG for aortic occlusion were categorized by whether or not aortic occlusion was manifested, and the correlation between maternal age, gender, diabetic malfunction, and kidney and liver abnormality and renal cysts was estimated. The correlation of clogged aorta was demonstrated by a multifactorial logistic regression with gender and the presence of renal cysts (*P* < 0.05); (3) the correlation of clogged aorta was demonstrated by a multifactorial logistic regression with renal cysts as an independent risk factor for clogged aorta (95% CI: 1.028–10.291;*P* = 0.031).

**Conclusion:**

As renal cysts are an autonomous risk of aortic coarctation, it is recommendable to strengthen clinical investigations such as monitoring of clinical blood pressures in kidney cyst recipients to assess their aortic function in order to evaluate their prognosis and minimize the prevalence of aortic coarctation.

## 1. Introduction

Aortic coarctation is a phenomenon in which blood from the lumen of the aorta passes through an endothelial breach and enters the middle layer of the aortic wall, thereby forming haematoma [1]. Aortic coarctation is not an expansion of the aortic wall and differs markedly from aortic aneurysm [2]. Aortic coarctation is currently one of the more common and most complex and dangerous cardiovascular diseases, with an incidence of approximately 100 per 100,000 people per year, and its incidence has tended to increase in recent years as the population's dietary habits and lifestyles have changed [3, 4].

Aortic coarctation is still a great challenge for clinicians. It is an acute vascular pathology that is associated with various pathologies such as hypertension, atherosclerosis, hyperlipidaemia, and Marfan syndrome. The study of these related diseases not only aids to reveal the pathogenesis of renal cysts but also has positive implications for predicting the emergence of aortic coarctation [5, 6]. In recent years, as research on aortic coarctation has intensified, some scholars have pointed out that renal cysts are more common in patients with aortic coarctation [7], but there are still few studies on the association between these two diseases. We now propose to analyse the association between aortic coarctation and renal cysts by including 244 patients with aortic coarctation as subjects, with the aim of contributing to the diagnosis and prognosis of these conditions.

## 2. Materials and Methods

### 2.1. General Data

Retrospectively, 244 patients with aortic coarctation who were undergoing inpatient treatment at our hospital from April 2014 to December 2021 were selected as the investigation category (study category, SG category), 150 patients with essential hypertension who consulted at our museum during the same period were the case-control category (matched category, MG category), and 150 healthy physical examiners were the control category (control category CG category). This research has been reported to the hospital ethics committee for approval.

#### 2.1.1. Inclusion and Exclusion Criteria for Patients in the SG Category

(1) All met the diagnostic criteria of the American Heart Association Guidelines for Aortic Coarctation [8] and were diagnosed under imaging; (2) clinical data were complete and available. Exclusion criteria: (1) patients with comorbid psychiatric disorders; (2) those with comorbid end-stage renal disease, hydronephrosis, or renal tumours; (3) other unresolved clinical investigators have been included.

#### 2.1.2. Inclusion and Exclusion Criteria for Patients in the MG Category

(1) All patients in the category met the diagnostic criteria for hypertension in the Guidelines for the Treatment of Hypertension [9]; (2) clinical data were complete and available. Exclusion criteria: (1) repeated hospitalisation; (2) incomplete clinical data; (3) concurrent end-stage renal disease, hydronephrosis, renal tumour, aortic coarctation, and aortic aneurysm; (4) other unresolved clinical investigators have been included.

#### 2.1.3. Inclusion and Exclusion Criteria for Patients in the CG Category

Inclusion criteria: healthy individuals who underwent screening at our medical screening centre. Exclusion criteria: patients with end-stage renal disease, hydronephrosis, renal tumour, aortic coarctation, and aortic aneurysm.

### 2.2. Intervention Method

The age, gender, previous medical history of hypertension, and diabetes were included, and the admission symptoms, blood pressure, heart rate, and ancillary tests (liver and kidney function tests) of the three categories of individuals were recorded.

All individuals were divided into aortic coarctation and nonaortic coarctation categories according to the presence or absence of aortic coarctation, and analyses were conducted on the univariate and multifactorial logistic influencing factors of aortic coarctation to investigate the correlation between aortic coarctation and renal cysts.

### 2.3. Statistical Methods

The data were analysed using SPSS 24.0 statistical software. The Kolmogorov–Smimov test was used to test the normality of quantitative data. The indicators conforming to the normal distribution were tested by independent samples *t*-test (two groups) or analysis of variance (three groups or more), and the SNK test was used for post hoc comparison, and the results were expressed as mean ± standard deviation. The indicators that did not conform to the normal distribution were tested by the Kruskal–Wallis rank sum test, and the results were expressed as the median and quartile. The chi-square test was used for between-group comparisons of qualitative data. Differences were considered statistically significant at *P* > 0.05.

## 3. Results

### 3.1. Generic Clinical Data Analysis of the Three Clusters of Sufferers

The clinical data such as gender, age, history of diabetes mellitus, abnormal liver function, abnormal kidney function, and renal cyst were carried out to facilitate interaction between the three clinical categories, and the general clinical data showed that, in terms of mean age, history of diabetes mellitus, abnormal liver function, and abnormal kidney function, they did not differ substantially from each other (*P* > 0.05) (Table 1 and Figure 1).

### 3.2. Univariate Analysis of Aortic Coarctation in the Three Categories of Patients

The 244 SG patients, 150 MG patients, and 150 CG patients enrolled were categorized according to the presence or absence of aortic coarctation, and analysis was carried out on the correlation between mean age, gender, history of diabetes, abnormal liver and kidney function, and renal cysts and aortic coarctation, which revealed that the univariate consequence of aortic coarctation was gender and the presence or absence of renal cysts (*P* < 0.05) (Table 2).

### 3.3. Multifactor Logistic Regression Analysis of Aortic Coarctation

The univariate factors of gender and renal cyst associated with aortic coarctation were assigned (male = 0; female = 1; presence of renal cyst = 0; absence of renal cyst = 1), and multifactorial logistic regression analysis was performed on the dependent variable in relation to aortic coarctation. The results demonstrated that renal cyst was an independent risk factor for aortic coarctation (*P* < 0.05) (Table 3).

## 4. Discussion

Aortic coarctation is a state in which blood in the aortic lumen enters the aortic mesentery from a tear in the aortic intima, causing the mesentery to split and expand in the direction of the long axis of the aorta forming a true/false separation of the two lumens of the aortic wall [10]. The peak age of onset of aortic coarctation is 50–70 years, with a male to female ratio of about 2–3:1. About 65%–70% of patients with aortic coarctation will die in the acute phase due to cardiac compression and arrhythmias, making early diagnosis and treatment of the condition very important [11,12].

The management of aortic coarctation is still one of the hotspots of clinical research, and current studies have shown that it is closely related to various diseases such as hypertension, atherosclerosis, Marfan syndrome, and aneurysm [13]. In recent years, several scholars from home and abroad have pointed out that renal cysts may be closely associated with aneurysms [14], while others have directly pointed out that aortic coarctation may be associated with renal cysts [15]. In this study, 244 patients with aortic coarctation were included and analysed, and the combined incidence of renal cysts in the enrolled patients was 27.05% (66/244), which far exceeded the 12.00% (18/150) in the MG category and 8.00% (12/150) in the CG category, which is similar to the findings of other scholars. A retrospective analysis of 405 patients with aortic coarctation noted that the prevalence of renal cysts in this category was 36.5%, and another study found that the prevalence of renal cysts in patients with aortic coarctation after receiving propensity matching was 37.00%, well above 9% in normal individuals [16].

The authors of this paper analysed that this result confirms that there may be a similar pathogenesis between aortic coarctation and renal cysts. Studies have confirmed that polycystin is an essential component in maintaining the body's structure and that this protein is extensively involved in processes such as cell contraction, proliferation, and apoptosis, as well as having a specific relationship with polycystic kidney disease [17]. It has been noted that polycystin 1 and polycystin 2 are two isoforms of polycystin with expressed genes PKD1 and PKD2, which have been shown to be key genes in the development and progression of cystic kidney disease [18]. An animal study found that if the PKD1 and PKD2 genes were knocked out in mice, a series of changes such as fibrous breaks in the vessel wall, varying degrees of haematoma, and even entrapment in the vessel wall were also observed in the model mice [19]. Another animal study found that PKD1 knockout mice expressed polycystin 1 at only 25% of the level of normal mice, and postmortem examination revealed that five of the nine knockout mice showed preaortic coarctation manifestations such as intravascular wall haematomas [20]. These measurements demonstrate that aortic coarctation and renal cysts have a similar pathogenesis, and that the presence of renal cysts may have an inhibitory factor on the immunity of the aortic coarctation.

Renal cysts are an independent risk element for aortic coarctation, and it is recommended that clinical investigations such as blood pressure monitoring in patients with renal cysts be strengthened to assess aortic fitness so as to assess aortic function in an attempt to optimise patient prognosis and minimize the incidence of aortic coarctation.

## Figures and Tables

**Figure 1:** Diagnosis of generic commercial statistics of the three clinical categories. In the three categories, the discrepancy in median age showed no statutory sensitivity (*P* > 0.05) (Figure (a)), while the variance on gender and prevalence of renal cysts was regarded as supplementary variance between categories (*P* < 0.05) (Figure (b)). #signifies a statistical sense of variance between categories for the identical index.

**Table 1:** Anatomy of the overall mechanical data of the victims in the corresponding categories.

General information	SG (*n* = 244)	MG (n = 150)	CG (n = 150)	*P* ^*a*^	*P* ^*b*^
Mean age (years)	54.16 ± 5.04	54.62 ± 5.66	54.74 ± 4.91	0.402	0.263
Male/female	136/39	90/60	87/63	0.032	0.019
History of diabetes mellitus	9	6	9	0.817	0.802
Abnormal liver function	15	12	6	0.970	0.365
Abnormal kidney function	18	12	18	0.737	0.237
Renal cysts	66 (27.05)	18 (12.00)	12 (8.00)	0.004	0.001

**Table 2:** Univariate analysis of aortic coarctation in the three categories of aortic coarctation.

Clinical characteristics		Aortic coarctation category (n = 244)	No aortic coarctation category (n = 300)	*t/X* ^*2*^	*P*
Mean age (years)		54.16 ± 5.04	54.69 ± 4.58	0.140	0.889

Gender	Male	136	177	17.224	<0.001
	Female	39	123		
History of diabetes	Yes	9	15	0.549	0.459
	No	235	285		

Abnormal liver function	Yes	15	18	0.005	0.943
	No	229	282		

Abnormal kidney function	Yes	18	30	1.151	0.283
	No	226	270		

Renal cysts	Yes	66	30	26.913	<0.001
	No	178	270		

**Table 3:** Multi-factor logistic regression thesis of aortic coarctation.

Variables	*β*	SE	Wald	95% CI	*P*
Gender	1.022	0.417	1.819	0.421–0.781	0.054
Renal cysts	1.698	0.851	0.071	1.084–10.5189	0.006

## Data Availability

All data generated or analysed during this study are included in this published article.
